The article "High-Concentration Metformin Reduces Oxidative Stress Injury and Inhibits the Growth and Migration of Clear Cell Renal Cell Carcinoma" was published in 2022. Journal: Comput Math Methods Med.

# High-Concentration Metformin Reduces Oxidative Stress Injury and Inhibits the Growth and Migration of Clear Cell Renal Cell Carcinoma

**DOI:** 10.1155/2022/1466991

**Published:** 2022-05-10

**Authors:** Yang Liu, Jianwei Li, Miaomiao Song, Guisong Qi, Lingling Meng

**Affiliations:** ^1^The Second Department of Urology, Cangzhou Central Hospital, China; ^2^The Third Department of Endocrinology, Central Hospital of Cangzhou, China

## Abstract

**Objective:**

To explore the mechanism of metformin in treating *CCRCC*.

**Methods:**

Prospective cohort study was conducted. *SOD* and *cyclin D* in six *CCRCC* samples donated by volunteers were detected to compare the degree of oxidative stress injury and the status of cell proliferation. *786-0 CCRCC* cells were cultured *in vitro* with different concentrations of metformin, and *MTT* assay and *Transwell* cell migration and wound healing assay were used to detect their proliferation and migration. After culture, *SOD* and *cyclin D* in *786-0 CCRCC* cells were also detected.

**Results:**

In the edge tissue, *SOD* was lower than in the tumor nest and normal tissue, and *cyclin D* was highly expressed. In grade *II CCRCC*, *SOD* was higher than in grade *IV CCRCC*, but *cyclin D* was also highly expressed in grade *IV CCRCC*. The cell proliferation rate and density of the metformin group were lower than the control group, while in the high-concentration metformin group, it was lower than medium- and low-concentration groups. After culture, the migration of *786-0* cells in the metformin group was significantly lower than that in the control group, the wound healing rate was decreased, and the migration and wound healing rates in the high-concentration metformin group were significantly lower than those in the medium- and low-concentration groups. However, the *SOD* of the metformin group was higher than the control group, but the *cyclin D* was lower, while the *SOD* was higher than medium- and low-concentration groups in the high-concentration group, but the c*yclin D* was lower after cultured.

**Conclusion:**

High-concentration metformin can reduce oxidative stress injury, increase the expression of *SOD* in *CCRCC*, and reduce *cyclin D* in *CCRCC* to inhibit proliferation and migration, which has optimistic prospects and application value in controlling the progression of *CCRCC*.

## 1. Introduction

Renal cell carcinoma (RCC) is a highly malignant tumor in the urinary system and one of the most common tumors. It is a malignant tumor originating from the renal parenchyma and urinary tubular epithelial system, also known as renal adenocarcinoma, accounting for 80%~90% of renal malignant tumors. According to the survey, renal cell carcinoma occupies the second place in China's urogenital tumors, second only to bladder tumors, accounting for 2%~3% of adult malignant tumors and about 20% of pediatric malignant tumors. There is a significant difference in incidence rate between men and women. According to statistics, the ratio of men to women is 2 : 1. The incidence of renal cell carcinoma increases with age. Data show that the incidence rate of renal cell carcinoma is 40~55 years old. In addition, the incidence of renal cell carcinoma has obvious international differences. The incidence rate of renal cancer is obviously higher in Europe and America than in Asian countries, and the incidence rate of cancer in Japan and India is low. The incidence rate of city is higher than that of rural area [1–5]. Although radical nephrectomy or nephron-sparing surgery could achieve 5-year disease-free survival for more than 90% of patients with localized renal cell carcinoma, there were still approximately 20%-30% recurrence and metastasis rates after surgery. Second, approximately 1/3 of renal cell carcinoma patients had been found to have metastasis at the first visit, so it was difficult to accept radical surgery [6, 7]. As a result, the prognosis of metastatic renal cell carcinoma (*mRCC*) is very poor, the median survival time is only 6-12 months, and the 5-year survival rate is less than 10% [8, 9]. Therefore, delaying the progression of renal cell carcinoma is still a major clinical challenge.

The article "High-Concentration Metformin Reduces Oxidative Stress Injury and Inhibits the Growth and Migration of Clear Cell Renal Cell Carcinoma" was published in 2022. Journal: Comput Math Methods Med.

Studies have found that patients who use metformin have a lower risk of cancer and lower cancer-related mortality [10, 11]. Some experimental studies have found that metformin can inhibit the proliferation of prostate cancer cells [12], breast cancer cells [13], pancreatic cancer cells [14], and melanoma cells [15] *in vitro*. Some *in vivo* experiments also confirmed that metformin could inhibit tumor growth [16, 17]. Therefore, metformin might have significance in the prevention and treatment of tumors.

However, there are few reports about the effect of metformin on the growth of renal cell carcinoma, especially the study of metastatic clear cell renal cell carcinoma (*CCRCC*). Whether metformin affects the proliferation, migration, and death of *CCRCC* and whether metformin inhibits the growth of *CCRCC* are also unknown.

Based on the above thinking, we detected and analyzed renal tissue samples of clear cell renal cell carcinoma and conducted cell experiments on *786-0* clear cell renal cell carcinoma cell lines *in vitro* to verify the relationship between metformin and the growth and migration of clear cell renal cell carcinoma. We found that metformin could reduce oxidative stress injury and inhibit the progression of renal cell carcinoma, which provided a new idea for the clinical treatment of renal cell carcinoma.

The article "High-Concentration Metformin Reduces Oxidative Stress Injury and Inhibits the Growth and Migration of Clear Cell Renal Cell Carcinoma" was published in 2022. Journal: Comput Math Methods Med.

## 2. Materials and Methods

### 2.1. Ethics

This study was approved by the ethics committee of *Cangzhou Central Hospital of Hebei Province*, and informed consent was obtained. The study was conducted in accordance with the Oxidative Medicine and Cellular Longevity policy for experimental and clinical studies [18].

### 2.2. Tissue Sample Study

Six cases of clear cell renal cell carcinoma (*CCRCC*) were collected and divided into three groups according to the different tissue structures, including 6 cases of cancer nest tissue, 6 cases of cancer nest edge tissue, and 6 cases of adjacent normal tissue.

#### 2.2.1. General Information

All patients were from the *Department of Urology*, *Guangdong Provincial People*'*s Hospital*. The average age was 55.67 ± 8.80 years (range, 43~67 years). The course of disease was 15.17 ± 7.14 months (range, 6~24 months).

#### 2.2.2. Classification

According to the 2016 version of the renal tumor classification standard [19] and 2012 *WHO/ISUP* classification system [20], combined with the 2020 “Chinese guidelines for the diagnosis and treatment of urology and andrology diseases” [21], the clinical classification and classification were carried out, including 1 case of *grade I*, 2 cases of *grade II*, 1 case of *grade III*, and 2 cases of *grade IV*.

#### 2.2.3. Inclusion Criteria

Inclusion criteria are as follows: ① according to the clinical diagnosis of renal cell carcinoma, the first diagnosis was renal cell carcinoma; ② be able to receive long-term follow-up and sign informed consent; ③ according to the indication of radical nephrectomy, informed consent was signed; and ④ can cooperate with surgical treatment.

#### 2.2.4. Exclusion Criteria

① They did not meet the inclusion criteria. ② Who could not cooperate with the corresponding examination and follow-up?.

### 2.3. Cell Experiment *In Vitro*

#### 2.3.1. Materials and Equipment

The human *786-0 CCRCC* cell line was purchased from the *Shanghai Cell Bank of the Chinese Academy of Sciences*, and fetal bovine serum, *DMEM*, and double antibody were obtained from HyClone Company of Australia. Metformin hydrochloride (trade name: gehuazhi, national drug approval word *h20023370*, aluminum plastic packaging, *10* tablets per plate, *2* plates per box, and specification: 0.5 g/tablet) was purchased from *Sino US Shanghai Squibb Pharmaceutical Co., Ltd*. The proliferation and migration of *786-0* cells were observed before culture and after culture within *24 hours*, *48 hours*, and *72 hours*.

The article "High-Concentration Metformin Reduces Oxidative Stress Injury and Inhibits the Growth and Migration of Clear Cell Renal Cell Carcinoma" was published in 2022. Journal: Comput Math Methods Med.

#### 2.3.2. Methods and Steps

*(1) Determination of Superoxide Dismutase (Cu ZnSOD)*. The pyrogallol autoxidation method was used. Under alkaline conditions, pyrogallol was autoxidized to citrinol. *O^2-^* was tracked by ultraviolet visible spectroscopy at a wavelength of 420 nm. Superoxide dismutase (*SOD*) catalyzes the disproportionation reaction of *O^2-^* to inhibit the autoxidation of pyrogallol. The inhibition rate of the pyrogallol autoxidation rate was calculated, which can reflect the content of *SOD* in the sample. The calculation formula is as follows:

(1) $$\begin{array}{c} \text{SOD}\left(U\cdot g^{-1}\cdot \text{FW}\cdot h^{-1}\right)=\frac{\left(A_{0}-A_{s}\right)\times V_{t}\times 60}{A_{0}\times 0.5\times FW\times V_{S}\times t}. \end{array}$$

In the formula, *A*_0_ is the absorbance of the control tube under light; *A*_*s*_ is the absorbance of the sample determination tube; *V*_*t*_ is the total volume of the sample extract (*ML*); *V*_*s*_ is the amount of crude enzyme solution (*ML*); *t* is the illumination time of the color reaction (*min*); FW is the fresh weight of the sample (*g*).

*(2) MTT Method*. *786-0* cells in good growth condition were seeded on *96*-well plates according to 2 × 10^3^/well, each well was 200 *μ*l, and *6* parallel wells were set in each group. After *24 hours* of culture, the cells were replaced with metformin-containing medium. After *48 hours* of culture, *20 μ*lmtt (2 mg/ml) was added to each well and incubated at *37*°C for *4* hours. The *MTT* solution was removed. Then, *150 μ*l dimethylsulfite (*DMSO*) was added to each well and vibrated on an oscillator for 10 minutes. After the crystal was completely dissolved, the absorbance value a (at *570* nm) was measured by enzyme-linked immunosorbent assay. The ratio of viable cells with different concentrations of metformin was analyzed. The cell survival rate was calculated as follows: cell survival rate = absorbance value of test group/absorbance value of control group × 100%.

*(3) Transwell Cell Migration Test*. ① The number of tumor cells in logarithmic growth phase was adjusted to 1 × 10^6^ cells/ml in 0.1% bovine serum albumin (*BSA*) *DMEM*. ② *One hundred* UL cells were inoculated in the upper Transwell chamber. Cells treated with *1.6*, *4.0*, and *10.0* mg*/ml* bsglee were added. The control group was supplemented with the same volume of serum-free *DMEM* medium, and each group was set with three chambers. ③ Add *500 μ*l DMEM containing *15%* calf serum to the lower chamber, and then, culture at 37°C and *5% CO^2^* for *24 hours*. The cells on the upper layer of the filter membrane were wiped off with a cotton swab, and the filter membrane was fixed with methanol for *5* minutes. ④ The cells were dyed with Giemsa dye for *15* min. ⑤ Under 100x light microscopy, the number of cells passing through the membrane in five different fields was selected, the average number of cells was calculated, and the migration ability of the drug to tumor cells was calculated according to the following formula. Migration inhibition rate = (1 − average number of migrating cells in the experimental group/average number of migrating cells in the control group) × 100%.

*(4) Scratch Healing Experiment*. *786-0* cells were inoculated into *6*-well plates, and each group of cells was cultured for *24* h. Then, a straight line was drawn in the culture plate with *a 1* ml sampling gun to form a cell-free “bare” area. The scraped cells were washed with *PBS*, and then, the cells were cultured in *10% FBS* medium containing *10* mm metformin (experimental group) and without metformin (control group) and incubated. The images were collected at *0*, *24*, *48*, and *72 hours*. The *NIS* elements software was used to measure the width of the “bare” area of the cells at the top, middle, and bottom of the scratch in the image, and the average value was calculated. The migration index (IM) was used to express the speed of cell migration. Im = 100%(G0 GT)/G0. G0 refers to the width of the “bare” area at the scratch when the image is collected immediately after the scratch (*0* h), and GT refers to the width of the “bare” area at the scratch when the image is collected after the scratch cell culture.

The article "High-Concentration Metformin Reduces Oxidative Stress Injury and Inhibits the Growth and Migration of Clear Cell Renal Cell Carcinoma" was published in 2022. Journal: Comput Math Methods Med.

### 2.4. qRT–PCR

#### 2.4.1. Sample Processing

*(1) Tissue*. The tissue was frozen at *-70°C*, 1 ml *TRIzol* reagent was added to every *30~50* mg of tissue, and the tissue was homogenized with a homogenizer. Then, they were divided into experimental groups (blank control group, cancer nest tissue groups, cancer nest edge tissue groups, and adjacent normal tissue groups). *RNA* was extracted from the tissues, and *cyclin D* in each sample was detected (*GAPDH* protein was used as an internal reference).

*(2) Cells*. Remove the culture solution from the culture bottle with a micro pipette, and add 1 ml of *4*°C precooled *PBS* solution, and shake and wash gently, and remove the *PBS* with a micro pipette. Add 1 *ml* of *TRIzol* reagent, shake gently, or blow with a gun head to break the cells. Cells in the logarithmic growth stage were collected, counted, resuspended in complete medium, the cell concentration was adjusted to 1 × 10^5^*cells/ml* and inoculated into *6-*well plates, and *2* ml of cell suspension was added to each well. After the cells adhered to the wall, they were divided into experimental groups (blank control group, low metformin concentration groups (*0.5* mmol*/L*), medium metformin concentration groups (*5 mmol/L*), and high metformin concentration group (*50* mmol*/L)*). *RNA* was extracted from the cells, and *cyclin D* in each sample was detected (*GAPDH* protein was used as an internal reference).

The article "High-Concentration Metformin Reduces Oxidative Stress Injury and Inhibits the Growth and Migration of Clear Cell Renal Cell Carcinoma" was published in 2022. Journal: Comput Math Methods Med.

#### 2.4.2. Reagent and Instrument

The reagent and instrument are shown in Tables 1 and 2.

#### 2.4.3. Quantitative PCR

The primer sequences are shown in Table 3, the *PCR* system is shown in Table 4, and the *PCR* amplification is shown in Table 5.

#### 2.4.4. Result Analysis

*ΔΔ* CT method

*A* = CT (target gene, sample to be tested) − CT (internal standard gene, sample to be tested).

*B* = CT (target gene, control sample) − CT (internal standard gene, control sample).

*K* = *A* − *B*.

Expression multiple = 2^−k^.

### 2.5. Western Blot

The tissues and the cultured cells were collected, and the concentrations of *cyclin D* in each sample were detected (*β*-actin protein was used as an internal reference) by *Western blot*. The specific steps include the following: ① protein extraction, ② protein concentration determination, ③ sample protein processing, ④ sample electrophoresis (Tables 6 and 7), ⑤ membrane transfer and immune reaction, ⑥ chemiluminescence color development, and ⑦ image analysis (ImageJ software processing).

### 2.6. Statistical Methods

*SPSS 19.0* and *GraphPad Prism 8.0* were used for statistical analysis and mapping. A *t*-test was used for the measurement data, a *chi-square* test was used for the count data, and *Pearson correlation analysis* was used for correlation analysis among various indicators. *P* < 0.05 was considered statistically significant.

## 3. Results

### 3.1. The *SOD* and *Cyclin D* in Tissues

The *SOD* in the edge tissue was lower than that in the tumor nest and adjacent normal tissue (Figure 1(a)), and in *grade II CCRCC*, it was higher than that in *grade IV* (Figure 1(b)). However, in the edge tissue, *cyclin D* was more highly expressed than in the tumor nest and adjacent normal tissue, while in grade *IV CCRCC*, it was also more highly expressed than grade *II* CCRCC (Figure 1(c)).

### 3.2. *MTT* Test Results

*786-0* cells were cultured with different concentrations of metformin for *72 hours*. The results showed that the cell proliferation rate of the metformin group was significantly lower than that of the control group, while the cell proliferation rate of the high-concentration metformin group was significantly lower than that of the medium-concentration and low-concentration groups (Figure 2).

### 3.3. *Transwell* Results

*786-0* cells were cultured with different concentrations of metformin. The results showed that the density of renal cancer cells in the metformin group was significantly lower than that in the control group, while the density of renal cancer cells in the high-concentration metformin group was significantly lower than that in the medium-concentration and low-concentration groups (Figure 3).

The article "High-Concentration Metformin Reduces Oxidative Stress Injury and Inhibits the Growth and Migration of Clear Cell Renal Cell Carcinoma" was published in 2022. Journal: Comput Math Methods Med.

### 3.4. *Wound Healing* Results

After culturing *786-0* cells with different concentrations of metformin for *24 hours*, the number of migrating cells in the metformin group was significantly lower than that in the control group, and the wound healing rate was significantly decreased. The cell migration and wound healing rates in the high-concentration metformin group were significantly lower than those in the medium-concentration and low-concentration groups (Figure 4).

### 3.5. *SOD* and *Cyclin D* in *786-0 Cells* after Cultured

*SOD* and *cyclin D* in *786-0 cells* after culture were detected. The results showed that the *SOD* of metformin group was significantly higher than control group, and in the high-concentration group, that was significantly higher than medium-concentration and low-concentration groups (Figure 5(a)). However, the *cyclin D* of the metformin group was significantly lower than the control group, and in the high-concentration group, that was significantly lower than medium-concentration and low-concentration groups (Figure 5(b)).

## 4. Discussion

In vivo free radicals refer to any molecule or ion containing one or more unpaired electrons. It is an intermediate product in the process of biochemical metabolism in vivo. It is considered a highly active chemical substance with active properties and strong oxidation ability that can regulate cell proliferation and apoptosis in two ways and affect a series of signal transduction pathways. First, a low concentration of superoxide anion free radicals (0-2) was necessary to maintain life, which could activate transcription factors and promote cell proliferation and differentiation; on the other hand, a high concentration of superoxide anion free radicals could cause oxidative damage to tissues and cells, leading to disease and even death. Under normal circumstances, the production and elimination of superoxide anion free radicals in the body were in dynamic balance. When the body was under excessive oxygen load, the formation of reactive oxygen species free radicals was too much, or the activity of antioxidant substances was decreased or even exhausted, which would cause the balance damage, oxidative stress state, cell *DNA* damage, and wrong repair that could lead to the activation of oncogenes or the inhibition of oncogenes or lead to cancer initiation. Recent studies found that free radicals were closely related to the occurrence and development of many diseases in the body [22, 23]. Some scholars found that in clinical practice, *ROS* levels were significantly increased in liver cancer, breast cancer, lung cancer, gastric cancer, and other malignant tumors [24–27]. Some studies have shown that oxidative stress could also promote the formation of tumor neovascularization and then promote the growth and metastasis of cancer masses [28, 29].

The article "High-Concentration Metformin Reduces Oxidative Stress Injury and Inhibits the Growth and Migration of Clear Cell Renal Cell Carcinoma" was published in 2022. Journal: Comput Math Methods Med.

There is a complete free radical scavenging system in the human body, including chemical scavengers and enzymatic scavenging systems. Chemical scavengers are natural scavengers, such as vitamin E, which widely exist in the body. These small molecules could block the peroxy free radical chain reaction through nonenzymatic reactions, prevent the oxidation and peroxidation of unsaturated fatty acids on the cell membrane, and protect cells from peroxide damage. The second was an enzymatic scavenging system, mainly including superoxide dismutase (*SOD*), glutathione peroxidase (*GSH-Px*), catalase, and other antioxidant enzymes, which removed excessive oxygen free radicals through specific enzymatic reactions. Superoxide dismutase (*SOD*) is an important antioxidant enzyme in the human body. There were five subtypes: *Cu ZnSOD*, *MnSOD*, *FeSOD*, *Ni SOD*, and *Fe ZnSOD*. *Cu ZnSOD* is a blue–green antioxidant enzyme that mainly exists in the cytoplasm of eukaryotic cells. Therefore, our study chose *Cu ZnSOD* as an index to evaluate the degree of oxidative stress injury in clear cell carcinoma renal tissue.

Recent studies have shown that *Cu ZnSOD* plays an important role in the occurrence and metastasis of non-small-cell lung cancer [30], gastric cancer [31], colon cancer [32], and liver cancer [33]. *Cu ZnSOD* could reduce the oxidative damage of cells and inhibit the invasion and progression of tumor cells. In this study, we also found that the *Cu ZnSOD* in the edge tissue was significantly lower than that in the tumor nest and adjacent normal tissue in one sample. Second, in different grades of *CCRCC*, *Cu ZnSOD* was also different; in grade *II* CCRCC, Cu ZnSOD was significantly higher than in grade *IV CCRCC*. It was suggested that the difference in oxidative stress injury was different in *CCRCC*. The possibility of cancer cell invasion was greater when oxidative stress injury was mild. At the same time, we detected the expression of *cyclin D* in different parts of the tissues to verify the growth of the cell cycle. We found that in the edge tissue, *cyclin D* was more highly expressed than in the tumor nest and adjacent normal tissue, while in grade *IV CCRCC*, it was also more highly expressed than grade *II CCRCC.* Therefore, we considered that improving the local oxygen free radical concentration and reducing oxidative stress injury might have important value in preventing cancer cells from invading normal tissues.

The article "High-Concentration Metformin Reduces Oxidative Stress Injury and Inhibits the Growth and Migration of Clear Cell Renal Cell Carcinoma" was published in 2022. Journal: Comput Math Methods Med.

Metformin is a noninsulin hypoglycemic drug that is widely used in the clinic. It could activate liver kinase, inhibit liver glycogenesis and fat synthesis, increase insulin-mediated glucose utilization, reduce insulin secretion of islets, or inhibit cholesterol biosynthesis and storage and had no obvious hypoglycemic effect on normal people. An epidemiological survey found that insulin resistance, hyperglycemia, and high insulin levels were risk factors for cancer [34]. Metformin could reduce the risk of these risk factors and reduce the risk of cancer. Small-scale studies have reported that patients using metformin have a lower risk of prostate cancer, breast cancer, liver cancer, and other tumors [35–37]. Some *in vitro* and animal experiments found that metformin could inhibit the proliferation and growth of prostate cancer cells, breast cancer cells, pancreatic cancer cells, and melanoma cells [38–41].

A retrospective cohort study on 84434 veterans found that in a 10-year retrospective analysis, metformin was not associated with most cancers, such as bladder cancer, breast cancer, colorectal cancer, esophageal cancer, gastric cancer, and prostate cancer, but there was a negative correlation with the liver, which might be helpful for the prevention of liver cancer [42]. Metformin has a certain effect on the proliferation and antimetastasis of human esophageal cancer cells *in vitro* [43]. This result suggested that renal cell carcinoma had nothing to do with the expression of insulin receptors, but metformin might reduce the level of hyperinsulinemia and inhibit the progression of renal cell carcinoma [44]. A previous study found that although obesity increased the risk of renal cell carcinoma, the survival time of obese patients with renal cell carcinoma was longer than that of nonobese patients. They found that metformin could induce tumor cell apoptosis through cell culture *in vitro* [45].

Combined with the detection results of clinical tissue samples of *CCRCC*, we carried out an *in vitro* culture experiment with *786-0* renal cell carcinoma cells. We found that the cell proliferation rate and density of the metformin group were lower than the control group, while in the high-concentration metformin group, it was lower than medium- and low-concentration groups. We performed two experiments to verify these results. First, the *MTT* and *Transwell* test results showed that the cell proliferation rate was significantly lower than that of the low-concentration group and the blank control group. Second, the wound healing test also confirmed that the number of migrating cells in the metformin group was significantly lower than that in the control group, and the wound healing rate was significantly decreased in the high-concentration metformin group compared with the medium-concentration and low-concentration groups. This was consistent with the research of other scholars, which indicated that in the process of proliferation and migration of *CCRCC*, reducing glucose concentration, reducing the energy supply required for cancer cell proliferation, and promoting cancer cells in a “hungry” state might be of great significance to slow down the proliferation of cancer cells.

The article "High-Concentration Metformin Reduces Oxidative Stress Injury and Inhibits the Growth and Migration of Clear Cell Renal Cell Carcinoma" was published in 2022. Journal: Comput Math Methods Med.

After culture, *SOD* and *cyclin D* in *786-0 cells* were also detected. This time is the *SOD.*

However, could low-glucose medium inhibit oxidative stress damage in cancer cells? Did metformin promote the self-protective function of cancer cells against oxidative damage *in vivo*? To confirm these findings, we detected the concentrations of *Cu ZnSOD* and *cyclin D* in *786-0 cells* after culture. The results showed that the *Cu ZnSOD* of the metformin group was significantly higher than the control group, and in the high-concentration group, that was significantly higher than medium- and low-concentration groups. However, the *cyclin D* of the metformin group was significantly lower, and in the high-concentration group, it was significantly lower. This verification led us to find that metformin could reduce the degree of oxidative stress injury, thereby inhibiting the number and growth rate of cancer cells, which might be one of the effective mechanisms of metformin in inhibiting renal cell carcinoma.

## 5. Conclusion

In conclusion, the degree of oxidative stress injury in different areas around the cancer nest was different in *CCRCC*, which was the most serious in the paracancerous tissues. High concentrations of metformin could effectively inhibit the proliferation and progression of the *786-0* renal cell carcinoma cell line by reducing oxidative stress injury and inhibiting the cell proliferation cycle in cancer tissues. High concentrations of metformin might have potential value in the treatment of *CCRCC*.

## Figures and Tables

**Figure 1:** The SOD and cyclin D in tissues.

**Figure 2:** MTT test results.

**Figure 3:** Transwell results.

**Figure 4:** Wound healing results.

**Figure 5:** SOD and cyclin D in 786-0 cells after culture.

**Table 1:** The reagent.

Reagent	Specifications	Serial number	Manufacturer
DMEM/F12 culture medium	BR	A4192001	Gibco
FBS	BR	10099133	Gibco
Trypsin	BR	1213981	Gibco
Hank's buffer	500 ml	PB180321	Procell
TRIzol reagent	BR	DP424	TIANGEN
Reverse transcription kit		DBI-2220	DBI
Fluorescent quantitative PCR detection kit		AOPR-1200	Genecopies
DEPC		V900882	Vetec
Absolute ethanol, isopropanol, chloroform	AR		China
Metformin hydrochloride	0.5 g	h20023370	Sino
MTT cell proliferation test kit	500 t	MT-06	DOJINDO
Cyclin D antibody	10 *μ*l	Ab273608	Abcam

The article "High-Concentration Metformin Reduces Oxidative Stress Injury and Inhibits the Growth and Migration of Clear Cell Renal Cell Carcinoma" was published in 2022. Journal: Comput Math Methods Med.

**Table 2:** The instrument.

Instrument name	Model	Manufacturer
Biological inverted microscope	CKX41	OLYMPUS
Cell incubator	HERAcell® 150i	Thermo Fisher
Centrifuge	ST16	Thermo Fisher
Microplate reader	Multiskan GO	Thermo Fisher
SW-CJ-1FD super clean workbench	SW-CJ-1FD	SUJING
Real-time PCR	7500	ABI
Micro nucleic acid quantizer	SMA4000	Merinton

**Table 3:** The primer sequences.

Gene name	Gene ID	Primer sequence (5′-3′)		Amplification length (bp)
h-GAPDH	NM_001289745.3	Forward	CAAGAGCACAAGAGGAAGAGAG	102
		Reverse	CTACATGGCAACTGTGAGGAG	
h-Cyclin D	NM_053056.3	Forward	GTTCGTGGCCTCTAAGATGAAG	76
		Reverse	GATGGAGTTGTCGGTGTAGATG	

**Table 4:** PCR reaction system.

2× all-in-one qPCR mix	10.0 *μ*l
PCR forward primer (2 *μ*M)	2.0 *μ*l
PCR reverse primer (2 *μ*M)	2.0 *μ*l
cDNA	2.0 *μ*l
50× Rox Reference Dye	0.4 *μ*l
ddH_2_O	3.6 *μ*l

**Table 5:** PCR amplification.

Cycles	Steps	Temperature	Time	Detection
1	Initial denaturation	95°C	10 min	No
40	Denaturation	95°C	10 s	No
	Annealing	55°C	20 s	No
	Extension	72°C	35 s	Yes

**Table 6:** Separating gel formula.

Separation gel concentration	8%	10%	12%	15%	18%	20%
H_2_O mL	4.63	4	3.3	2.3	1.3	0.63
30% acrylamide (29 : 1) mL	2.67	3.3	4	5	6	6.67
1.5 M Tris-HCl (pH 8.8) mL			2.5 mL			
10%SDS mL			0.1 mL			
AP mL			0.1 mL			
TEMED *μ*L			5 *μ*L			
Total volume mL			10 mL			

**Table 7:** Concentrated gel formula.

Reagent	5% concentrated glue			
H_2_O mL	2	3	4	6
30% acrylamide (29 : 1) mL	0.5	0.75	1	1.5
1 M Tris-HCl (pH 6.8) mL	0.5	0.75	1	1.5
10%SDS *μ*L	40	60	80	120
AP *μ*L	30	45	60	90
TEMED *μ*L	4	6	8	12
Total volume mL	3	4.5	6	9

## Data Availability

The datasets generated during and/or analyzed during the current study are available from the corresponding author on reasonable request.
